# High Seroprevalence of Hepatitis B and C Virus Infections among Pregnant Women Attending Antenatal Clinic in Borumeda General Hospital, Northeast Ethiopia

**DOI:** 10.1155/2022/1395238

**Published:** 2022-08-28

**Authors:** Daniel Gebretsadik, Minilik Assefa, Genet Molla Fenta, Chala Daba, Abdurrahman Ali, Saba Gebremichael Tekele

**Affiliations:** ^1^Department of Medical Laboratory Science, College of Medicine and Health Sciences, Wollo University, P.O. Box 1145, Dessie, Ethiopia; ^2^Department of Environmental Health Science, College of Medicine and Health Sciences, Wollo University, Dessie, Ethiopia

## Abstract

**Background:**

Viral hepatitis are considered as the cause of solemn health problem for the human kind, particularly among pregnant women in the 21^th^ century. Therefore, this study is aimed at determining the seroprevalence of HBV and HCV infection among pregnant women attending at Borumeda General Hospital, Dessie, Northeast Ethiopia.

**Methods:**

An institution-based cross-sectional study was conducted at Borumeda General Hospital from April to May, 2020. A consecutive total of 124 pregnant women who were attending at the antenatal clinic (ANC) of the hospital were included. A structured questionnaire was used to assess the associated factors and some sociodemographic characteristics. Five milliliters of venous blood was collected from each study participant, and a laboratory test using a rapid HBsAg and anti-HCV kit was done. The data were analyzed using SPSS software version 22.

**Results:**

The mean age of the study subjects was 25.81 (*±*5.967) years. The overall seroprevalence of either HBV or HCV infections among the study participants was 14 (11.3%). HBsAg and anti-HCV were positive among 10 (8.1%) and 4 (3.2%) study participants, respectively. There was no coinfection result between HBV and HCV among pregnant women. Pregnant women who had abortion history [AOR 5.723; 95% CI 1.100-29.785, *P* value = 0.038] and hospitalization history with IV medication [AOR 6.939; 95% CI 1.017-47.322, *P* value = 0.048] exhibited statistically significant association with HBV infection.

**Conclusions:**

Seroprevalence of HBV and HCV infections among pregnant women was high, and the rate of HBV particularly can be considered in the high endemic category of the WHO classification scheme. Continuous screening of pregnant mothers, provision of hepatitis B vaccine for females at the child-bearing age, and health education to create awareness about HBV and HCV should be implemented.

## 1. Background

Viral hepatitis is challenging the health condition of the people around the world and considered the cause of solemn health problem for the human kind in the 21^th^ century [1–3]. In the globe, there are two well-known forms of chronic hepatitis, and this corresponds to hepatitis B virus (HBV) and hepatitis C virus (HCV). According to the World Health Organization (WHO) report, in the year 2019, there were 1.5 million new cases of chronic hepatitis B and C infection each in the globe [4]. The overall prevalence of HBV among general population and blood donors in 13 European Union countries between the years 2005 and 2015 was 0.9%; besides, this report also showed a slightly higher rate of HCV [5].

HBV and HCV can be prevalent and affect a wide range of population that includes human immunodeficiency virus- (HIV-) infected individuals, health care workers, blood donors (general population), pregnant mothers, and their children [3, 5–7]. Various studies indicate that the prevalence of HBV and HCV among pregnant women becomes serious public health importance [7–9]. Mother-to-child transmission of HBV, which might be via intrauterine transmission, is a common phenomenon and causes chronic infection of the virus [10]. The seroprevalence of HBV among pregnant women in Ethiopia ranges from 4.5% to 7.9%, that is in line with intermediate level of endemicity of the virus [11–15]. In most studies done in Ethiopia, the seroprevalence of HCV was lower than HBV and it ranges from 0.26% to 8.07% [9, 15–17].

Various factors are responsible for the seroepidemiology of HBV and HCV among pregnant women. The seroprevalence of HBV infections is affected by factors like having history of poly-sexual practices, previous history of dental procedures, health facility admission, genital mutilation, history of abortion, home delivery by traditional birth attendants, and blood transfusion [12, 15, 17, 18]. Some studies about the associated factors of HCV among pregnant women also revealed different determinants influence the seroepidemiology of the virus. A study conducted in Pakistan showed a history of surgical procedure, and maternal age determines the prevalence of HCV [19]. Even though it is not statistically supported, the prevalence of both HBV and HCV was higher among pregnant women who are living in the rural area [19–21].

So far, various studies regarding the seroprevalence of the two major causative agents of viral hepatitis (HBV and HCV) with their associated factors among pregnant women were done. Majority of these studies were conducted in health care facilities that serve urban resident populations. In Amhara region particularly in Dessie town, there is paucity of research output that shows the seroprevalence and determinant factors of HBV and HCV among pregnant women. In addition, the COVID-19 pandemic imposes paramount effect on the health care system and health care facilities like ANC service in different localities. Conducting such study in order to fill the literature gap that exists in the study area and to provide pertinent information for the policy-makers and researchers particularly in semiurban and rural set-up is highly important. So, this study was conducted to determine the seroprevalence and associated factors of HBV and HCV among pregnant women at Borumeda General Hospital in the era of COVID-19.

## 2. Methods

### 2.1. Study Area, Design, and Period

A hospital-based cross-sectional study that is aimed at investigating the prevalence and associated factors of HBV and HCV among pregnant women was conducted at Borumeda General Hospital from April to May, 2020. Borumeda General Hospital was established in 1947 EC through the support of a missionary organization that was primarily focused on dermatology and ophthalmic services. The hospital has long-time experience in dermatology and ophthalmology services. Currently, Borumeda General Hospital provides comprehensive health services, including antenatal care, medical, surgical, psychiatric clinic, and leishmaniasis for urban, semiurban, and rural residents. Since the hospital is located in a rural area in Dessie town, the majority of antenatal care service seekers were employed in the nearby localities.

### 2.2. Study Population

The study population recruited in this study was all pregnant women who visited the ANC clinic of Borumeda General Hospital during the data collection period and who fulfilled the inclusion criteria. Pregnant women with critical sickness and unable to give consent were excluded from the study. In order to have a representative sample of the pregnant women, the sample size was determined using a single population proportion formula. By considering the 4.9% previous prevalence with 4% margin of error (*d* = 0.04) and 95% confidence level (*Z*_*α*/2_ = 1.96). Then, computing with this formula and after applying 10% nonresponsive rate, the final sample size became 124. The consecutive sampling technique was used to recruit study participants.

### 2.3. Data Collection

#### 2.3.1. Sociodemographic/Clinical Data Collection

Sociodemographic characteristics of pregnant women (such as age, resident, marital status, educational level, occupational status, trimester, and gravidity) and also clinical data were collected consecutively from people who were enrolled for ANC follow-up at Borumeda General Hospital by using a structured questionnaire via face to face interview.

#### 2.3.2. Blood Sample Collection and Processing

Five milliliters of venous blood was collected from each study participant through vein puncture, dispensed with serum glass tubes; we waited 20-30 minutes for fibrin formation and then let the sample centrifuge at a relative centrifugal force of 1000-1500 g for 10 minutes, following standard operational procedures (SOPs). The serum was stored in a colder state until ready for a test. Positive and negative control samples within the test kits were run to assess the performance of the test kits. All laboratory procedures were carried out using SOPs. In preanalytical procedures, an adequate blood sample was collected carefully, and a labeled, dried, and leak-proof tube was used. In analytical blood examination, all collected serum specimens were tested with separate kits for HBsAg and anti-HCV antibody using rapid diagnostic test kits according to the manufacturer's guidelines (EUGENE HBsAg/HCV antibody rapid test, Shanghai Eugene Biotech Co., Ltd.).

#### 2.3.3. Data Quality Management

The quality of data was assured by properly designing the instrument for its simplicity and by recording all necessary data in predesigned questionnaire and formats. Pretests were done at 5% of the sample size at Dessie health center. Then, based on the findings of the pretests, necessary corrections and modifications have made to the questionnaire. The questionnaire was first prepared in English and converted to Amharic version and then converted to the English version for analysis. During data collection, proper categorization and coding of questionnaires and formats are made, and then the data is checked carefully on a daily basis for its completeness, consistency, and clarity. All the required materials and reagents (rapid HBsAg, anti-HCV antibody test kits, glass tubes, and 70% alcohol) were checked by quality control measurements.

#### 2.3.4. Data Analysis Procedures

The collected data were entered into EpiData and exported to SPSS version 22.0 statistical software for data clearing, coding, and analysis. Descriptive statistics like frequencies, standard deviation (SD), and percentage were done to summarize the data. Bivariable and multivariable logistic regression analyses were also used to investigate the statistical significance between the participant characteristics [both sociodemographic characteristics and clinical risk factors] and outcome variables (HBsAg and anti-HCV antibody positivity). AOR along with 95% CI was used to check the strength of association. Thus, a *P* value of <0.05 was used to cut the statistical significance point of the variables.

## 3. Results

### 3.1. Sociodemographic and Clinical Characteristics

A total of 124 pregnant women were included for screening. The mean age of the study subjects was 25.81 years with a standard deviation of *±*5.967 years. Almost half of the study subjects (72 (58.1)) were in the age group of 25 years and below, while the rest (52 (41.9)) were from 26 up to 45-year-old category. From the total participants, 114 (91.9%) were married and 51 (41.1%) were attending primary school or elementary school. Gravidity status showed that about 72 (58.1%) were primigravida and 52 (41.9%) had a previous delivery history (multigravida). Regarding occupational status, out of 124 pregnant women, 83 (66.9%) were house wives (Table 1).

### 3.2. Prevalence of HBV and HCV Infection

The overall seroprevalence of either HBV or HCV among the study participants was 14 (11.3%). Specifically, HBsAg and anti-HCV were positive among 10 (8.1%) and 4 (3.2%) study participants, respectively. In the present study, there was no coinfection result between HBV and HCV among pregnant women. From 72 (58.1%) pregnant women whose age was less than 25 years, 6 (8.3%) were positive for HBsAg and 3 (4.2%) for anti-HCV antibody. The prevalence of HBV infection was found relatively lower among rural dwellers. Eight of the one hundred fourteen married women were positive for HBsAg; 3 (2.6%) were positive for ant-HCV antibody (Table 1).

### 3.3. Prevalence and Associated Factors with HBV and HCV Infections

Exposure to different risk factors for HBV and HCV infection was assessed and investigated in this study. From 17 (62.9%) pregnant women who had a hospital admission history, 5 (29.4%) and 1 (5.9%) were infected with HBV and HCV infection, respectively. Out of the total study participants who had a history of either minor or heavy surgery, 6 (18.2%) were positive for HBsAg and 1 (4.5%) was infected by HCV infection. Among fifteen pregnant women who had multiple sexual partners, 5 (33.3%) were infected by HBV and 3 (20.0) by HCV. Out of six pregnant women who had a history of blood transfusion, 3 (50%) were positive for HBV infection and 1 (16.7%) was for HCV. From a total respondents, 15 pregnant women had abortion history; out of these, 4 (26.9%) were positive for HBsAg and 2 (13.3%) for anti-HCV antibody (Table 2).

Both bivariable and multivariable logistic regressions were done to assess the variables in relation to both HBV and HCV infections among pregnant women. In bivariable logistic regression analysis, pregnant women who had a history of surgical procedure, abortion history, a history of blood transfusion, and a history of multiple sexual partners and have multiple sexual partners without using a condom showed association with HBV infection and progressed to multivariable regression. But in the multivariable logistic regression, only two variables were found to be statistically significant. These variables were pregnant women who had abortion history [AOR 5.723; 95% CI: 1.100-29.785, *P* value = 0.038] and who had hospitalization history with IV medication [AOR 6.939; 95% CI: 1.017-47.322, *P* value = 0.048] (Table 3).

Moreover, with the same cut value, those with abortion history and having a history of multiple sexual partners, habit of drinking alcohol, and multiple sexual partners without using a condom proceed to multivariable logistic regression analysis of HCV infection, but there were no significant variables with anti-HCV antibody even though there were predictor variables from bivariable analysis (Table 4).

The logistic regression analysis of variables with the seroprevalence of either HBV or HCV showed only the history of abortion demonstrating significant association. Study participants who had history of abortion exhibited more than 11 times (AOR = 11.069, 95%CI = 1.465-83.599, *P* = 0.02) the likelihood of acquiring infection by the two common viral hepatitis types (Table 5).

## 4. Discussion

In the era of COVID-19 and other chronic infectious diseases like HIV, TB, and malaria, the disease pattern of viral hepatitis, particularly HBV and HCV in urban, semiurban, and rural set-ups, did not attract much attention. In some situations, even pregnant women may not be aware of their HBV serostatus [22], and only a few of the study participants had knowledge about HCV and HBV [23]. The two viral hepatitis seroprevalences among pregnant women become increased through the course of time in different localities of Ethiopia and various parts of Africa [6, 23–26]. On the contrary, viral hepatitis showed a decreasing pattern in certain developed countries like China [27]. A study was conducted comparing the seroprevalence of HBV and HCV among pregnant mothers inhabiting in rural and urban areas, and it was revealed that rural inhabitants were a highly affected group by these infections [28]. Similarly, a study, conducted in Ethiopia in which majority (80%) of study participants were urban dwellers, showed lower rate of infectivity to HBV and HCV [29]; other studies indicated that the prevalence of HBV and HCV was more common among rural area residents [9, 29, 30].

The overall seroprevalence of HBV and HCV among pregnant women in the current study was found to be 14 (11.3%). This rate of infection was higher than those in studies conducted in the northwestern part of Ethiopia and in Pakistan [17, 19]. A study conducted in Egypt indicated that only 1.2% of pregnant women were found to be infected with either HBV or HCV [7], whereas a study conducted in East Wollega, Ethiopia, showed comparable results in which 10.2% of study participants were infected with either HBV or HCV [9]. The discrepancy across these studies might be due to cultural and behavioral differences, sample size, and methodology.

The seroprevalence of HBsAg in the current study was 8.1% (10/124), and this rate of infectivity can be considered a highly endemic scenario of the virus [31]. The seroprevalence of HBsAg in the present study was comparable with other similar studies conducted in Ethiopia [18, 26, 32]. A cross-sectional study in Tanzania also reported consistent HBV infection rates among pregnant women [33]. Some other research findings in Ethiopia and abroad revealed that the seroprevalence of HBV among the same study subjects was lower than that of the current study [6, 13, 19, 20, 34]. On the contrary, some other studies showed higher HBV infection rate among different population groups and among pregnant mothers. A systematic review and meta-analysis report in Nigeria showed a higher rate (13.6%) of HBV among different populations in comparison with the current study. This report also indicated that the pooled prevalence of HBV among Nigerian pregnant women was found to be 14.1% [35]. Other studies which were conducted in Southern Ethiopia (10.9%) [36], Uganda (11.8%) [37], Cameroon (10.78%) [25], and the republic of South Sudan (11%) [38] showed slightly higher HBV infection rates. This variation in the seroprevalence of HBV among pregnant women might be due to differences in a study period, sample size, demographic characteristics, and other clinical conditions of the study participants across various localities.

Like those of most other similar studies [5, 39, 40], the seroprevalence of HBV among pregnant mothers in the present study was higher than that of HCV (8.1% versus 3.2%). In contrast to this, a study conducted in West Oromia, Ethiopia, showed higher HCV rate (8.07%) among pregnant women [9]. Another similar study in the Democratic Republic of Congo also showed a slightly higher HCV rate of infectivity (4.8%) than HBV (3.9%) [23]. In Egypt, even though the prevalence was very low, HCV was still indicated as the dominant infection over HBV [7]. This dominance of HCV over HBV in other studies might be associated with a nondetection ability of HBsAg due to mutation on the surface antigen gene [41].

The seroprevalence of HCV among pregnant women in the present study was higher than a systematic review of pooled prevalence in Ethiopia, whereas it was consistent with a subgroup analysis in Oromia region [16] and with a study conducted in Nigeria [42]. More than twofold rate of HCV positivity in comparison with the present study was demonstrated in a study conducted in Ghana [43].

In the present study, there were no any study participants who were infected with both of these viruses. A similar scenario in which the absence of HBV and HCV coinfectivity was documented in a lot of research work [17, 19, 44, 45]. Some other similar studies showed slight coinfectivity rate between the two viruses [43], and still, there are very few studies that indicate high rate of coinfectivity [42]. A study conducted in China explained about HCV spontaneous clearance among HBV/HCV-coinfected study subjects, and it also showed that female gender, concentration of HBV DNA, and genotype are associated with increased spontaneous clearance of HCV [46].

It was revealed that the history of hospitalization and history of abortion were strong predictor variables for HBV infection among pregnant women in the present study. Study participants with a history of hospital admission (IV medication) had 7 times the odds of acquiring HBV infection in comparison with their counterparts. Having a history of abortion had 5.7 times the likelihood of infection with HBV in relation with those study participants who did not have the history. Like those in the current study, both variables are indicated as having significant association with HBV infection in a study held in Southern Ethiopia [47]. In agreement with the present study, the history of abortion was mentioned as one of the predictor variables for HBV infection in studies conducted in Ethiopia [30, 48]. Some similar studies were inconsistent with the current study in which these two variables did not exhibit any association with HBV infection [34, 49]. A health facility study in Ethiopia indicated that the rate of HBV among abortion seeking young women was 1.94% [50]. According to UNFDP 2012 report, in Ethiopia, there was high abortion rate and low contraceptive utilization in women aged from 15 to 24 years [51]. The reason for abortion among females at reproductive age was unwanted pregnancy due to unsafe sexual practice [52, 53]. This unsafe sexual practice makes the women at risk of acquiring HBV and other STIs [54].

Like most studies conducted in Ethiopia and elsewhere, the present study did not only show statistically significant association between history of abortion and HCV infection [9, 55]. On the contrary to these studies, another study revealed association of HCV infection with a history of abortion [56]. This disparity could be due to the difference in laboratory diagnosis method, sample size, and demographic variation.

## 5. Limitation of the Study

The present study was conducted to provide epidemiological information about HBV and HCV infections among pregnant women in health facility which majorly provides health care (including ANC) for rural residents. But the study has limitation in relation with sample size, laboratory methods to screen HBV and HCV, and the number of health facility addressed. Even though we have calculated the determination of minimum sample size using single population proportion formula and it is representative of the source population, but still, the sample size is small.

## 6. Conclusions

In the current study, the seroprevalence of the two common viral hepatitis infections was high, and the rate of HBV particularly can be considered in the high endemic category of the WHO classification scheme. In order to reduce the prevalence of infections among pregnant women, a collaborative work among different stakeholders is mandatory. Continuous screening of pregnant mothers, provision of Hepatitis B vaccine for females at the child-bearing age, and health education to create awareness about HBV and HCV should be implemented. Having previous hospital admission history with IV medication and history of abortion were the determinant factors for the prevalence of HBV among pregnant mothers, whereas seroprevalence of HCV did not show any statistical significant association with the determinant variables. Proper care for hospital admitted patients, particularly for IV system medication administered patients, should be given. The health care service providers should consider their staffs to take continuous practical training on infection prevention methods. The possible reason for abortion needs to be supported by critical research works, and proper intervention like health education about the causes and effect of abortion should be provided. Routine antenatal screening for HBV and HCV infections during early pregnancy should be considered in order to control and prevent the possible vertical transmission of these viral agents. Furthermore, we recommend studies to be conducted to compare the real infections of HBV and HCV by using more advanced laboratory techniques among pregnant women living in rural and urban areas of Ethiopia.

## Figures and Tables

**Table 1:** Seroprevalence of HBV and HCV with sociodemographic characteristics among pregnant women attending antenatal care at Borumeda General Hospital from April to May, 2020 (*N* = 124).

Variables	Categories	Total Frequency (%)	HBV Frequency (%)		HCV Frequency (%)		HBV or HCV Frequency (%)	
			Positive	Negative	Positive	Negative	Positive	Negative
Age (years)	15-25	72 (58.1)	6 (8.3)	66 (91.7)	3 (4.2)	69 (95.8)	9 (12.5)	63 (87.5)
	26 & above	52 (41.9)	4 (7.7)	48 (92.3)	1 (1.9)	51 (98.1)	5 (9.6)	47 (90.4)

Residence	Urban	72 (58.1)	6 (8.3)	66 (91.7)	1 (1.4)	71 (98.6)	7 (9.7)	65 (90.3)
	Rural	52 (41.9)	4 (7.7)	48 (92.3)	3 (5.8)	49 (94.2)	7 (13.5)	45 (86.5)

Marital status	Married	114 (91.9)	8 (7.0)	106 (93.0)	3 (2.6)	111 (97.4)	11 (9.6)	103 (90.4)
	Single	10 (8.1)	2 (20)	8 (80)	1 (10)	9 (90)	3 (30)	7 (70)

Educational status	Secondary & above	27 (21.8)	3 (11.1)	24 (88.9)	1 (3.7)	82 (98.8)	4 (14.8)	23 (85.2)
	1-8	51 (41.1)	3 (5.9)	48 (94.1)	1 (2.0)	50 (98)	4 (7.8)	47 (92.2)
	Read & write	23 (18.5)	1 (4.3)	22 (95.7)	1 (4.3)	22 (95.7)	2 (8.7)	21 (91.3)
	Illiterate	23 (18.5)	3 (13)	20 (87)	1 (4.3)	22 (95.7)	4 (17.4)	19 (82.6)

Occupational status	Gov. employed	19 (15.3)	3 (15.8)	16 (84.2)	1 (5.3)	18 (94.7)	4 (21.1)	15 (78.9)
	Merchant	10 (8.1)	2 (20)	8 (80)	1 (10)	9 (90)	3 (30)	7 (70)
	Student	12 (9.7)	1 (8.3)	11 (91.7)	1 (8.3)	11 (91.7)	2 (16.7)	10 (83.3)
	House wife	83 (66.9)	4 (4.8)	79 (95.2)	1 (1.2)	82 (98.8)	5 (6)	78 (94)

Trimester	3^rd^	33 (26.6)	3 (9.1)	30 (90.9)	0 (0.00)	33 (100)	4 (11.8)	30 (88.2)
	2^nd^	44 (35.5)	2 (4.5)	42 (95.5)	0 (0.00)	44 (100)	3 (6.7)	42 (93.3)
	1^st^	47 (37.9)	5 (10.6)	42 (89.4)	4 (8.5)	43 (91.5)	7 (15.6)	38 (84.4)

Gravidity	Primigravida	72 (58.1)	4 (5.6)	68 (94.4)	2 (2.8)	69 (97.2)	6 (8.5)	65 (91.5)
	Multigravida	52 (41.9)	6 (11.5)	46 (88.5)	2 (1.9)	51 (96.2)	8 (15.1)	45 (84.9)

Previous place of delivery	No birth	70 (56.5)	4 (5.7)	66 (94.3)	2 (2.9)	68 (97.1)	6 (8.6)	64 (91.4)
	Health institution	33 (26.6)	3 (9.1)	30 (90.9)	1 (3)	32 (97)	4 (12.1)	29 (87.9)
	Home	21 (16.9)	3 (14.3)	18,(85.7)	1 (4.8)	20 (95.2)	4 (19)	17 (81)

**Table 2:** Seroprevalence of HBsAg and anti HCV antibody with risk factors among pregnant women attending antenatal care at Borumeda General Hospital from April to May, 2020 (*N* = 124).

Variables	Categories	Total Frequency (%)	HBV Frequency (%)		HCV Frequency (%)		HBV or HCV Frequency (%)	
			Positive	Negative	Positive	Negative	Positive	Negative
Hospitalization with IV medication	Yes	17 (13.7)	5 (29.4)	12 (70.6)	1 (5.9)	16 (94.1)	6 (35.3)	11 (64.7)
	No	117 (86.3)	5 (4.7)	102 (95.3)	3 (2.8)	104 (97.2)	8 (7.5)	99 (92.5)

Surgical procedures	Yes	22 (17.7)	4 (18.2)	18 (81.8)	1 (4.5)	21 (95.5)	5 (22.7)	17 (77.3)
	No	102 (87.3)	6 (5.9)	96 (94.1)	3 (2.9)	99 (97.1)	9 (8.8)	93 (91.2)

Abortion history	Yes	15 (12.1)	4 (26.9)	11 (73.3)	2 (13.3)	13 (86.7)	6 (40)	9 (60)
	No	109 (87.9)	6 (5.5)	103 (94.5)	2 (1.8)	107 (98.2)	8 (7.3)	101 (92.7)

History of blood transfusion	Yes	6 (4.8)	3 (50)	3 (50)	1 (16.7)	5 (83.3)	4 (66.7)	2 (33.3)
	No	118 (95.2)	7 (5.9)	111 (94.1)	3 (2.5)	115 (97.5)	10 (8.5)	108 (91.5)

Multi sexual partner	Yes	15 (12.1)	5 (33.3)	10 (66.7)	3 (20.0)	12 (80)	8 (53.3)	7 (46.7)
	No	109 (87.9)	5 (4.6)	104 (95.4)	1 (0.9)	108 (99.1)	6 (5.5)	103 (94.5)

Condom usage	No	111 (89.5)	6 (5.4)	105 (94.6)	2 (1.8)	109 (98.2)	103 (92.8)	8 (7.2)
	Yes	13 (10.5)	4 (30.8)	9 (69.2)	2 (15.4)	11 (84.6)	6 (46.2)	7 (53.8)

Sharing of sharp materials	Yes	74 (59.7)	6 (8.1)	68 (91.9)	3 (4.1)	71 (95.9)	9 (12.2)	65 (87.8)
	No	50 (40.3)	4 (8)	46 (92)	1 (2)	49 (98)	5 (10)	45 (90)

Ear and nose piercing	Yes	61 (49.2)	4 (6.6)	57 (93.4)	3 (4.9)	58 (95.1)	7 (11.4)	54 (88.6)
	No	63 (50.8)	6 (9.5)	57 (90.5)	1 (1.6)	62 (98.4)	7 (11.1)	56 (88.9)

Drinking of alcohol	Yes	29 (23.4)	4 (13.8)	25 (86.2)	3 (10.3)	20 (89.7)	7 (24.1)	22 (75.9)
	No	95 (76.6)	6 (6.3)	89 (93.7)	1 (1.1)	94 (98.9)	7 (7.4)	88 (92.6)

**Table 3:** Seroprevalence of HBV with their sociodemographic characteristics and risk factors among pregnant women attending antenatal care at Borumeda General Hospital from April to May, 2020 (*N* = 124).

Variables	Categories	COR [95% CI]	*P* value	AOR [95% CI]	*P* value
Age (year)	15-25	1.00		—	—
	26 and above	0.917 (0.245-3.427)	0.897	—	—

Residence	Urban	1.00		—	—
	Rural	1.091 (0.292-4.078)	0.897	—	—

Marital status	Married	1.00		—	—
	Single	3.312 (0.600-18.278)	0.169	—	—
	Widowed	—	—	—	—
	Divorced	—	—	—	—

Educational status	Secondary & above	1.00		—	—
	Primary (1–8)	3.300 (0.317-34.3543)	0.318	—	—
	Read & write	1.3750 (0.135-13.974)	0.788	—	—
	Illiterate	2.750 (0.266-28.433)	0.834	—	—

Occupational status	Gov. employed	1.00		—	—
	Merchant	1.795 (0.184-17.558)	0.615	—	—
	Student	4.937 (0.779-31.295)	0.090	—	—
	House wife	3.703 (0.755-18.168)	0.107	—	—

Trimester	3^rd^	1.00		—	—
	2^nd^	0.481 (0.076-3.050)	0.437	—	—
	1^st^	1.292 (0.286-5.825)	0.739	—	—

Gravidity	Primigravida	1.00		—	—
	Multigravida	2.138 (0.572-7.996)	0.259	—	—

Previous place of delivery	No birth	1.00		—	—
	Health institution	0.600 (0.109-3.296)	0.557	—	—
	At home	0.364 (0.075-1.774)	0.211	—	—

Hospitalization- IV medication	Yes	8.500 (2.146-33.664)	0.002	6.939 (1.017-47.322)	0.048^∗∗^
	No	1.00		—	—

Surgical procedures	Yes	3.556 (0.911-13.876)	0.068	0.548 (0.059-5.122)	0.598
	No	1.00			

Abortion history	Yes	6.242 (1.525-25.560)	0.011	5.723 (1.100-29.785)	0.038^∗∗^
	No	1.00			

Blood transfusion	Yes	15.857 (2.692-93.397)	0.002	1.980 (0.131-29.934)	0.622
	No	1.00			

Multi sexual partner	Yes	0.096 (0.024-0.390)	0.001	0.136 (0.002-10.419)	0.368
	No	1.00			

Condom usage	No	7.778 (1.849-32.719)	0.005	1.320 (0.017-102.083)	0.900
	Yes	1.00			

Sharing of sharp materials	Yes	1.015 (0.271-3.796)	0.983	—	—
	No	1.00		—	—

Ear and nose piercing	Yes	1.500 (0.402-5.600)	0.546	—	—
	No	1.00		—	—

Drinking of alcohol	Yes	2.373 (0.621-9.070)	0.206	—	—
	No	1.00		—	—

∗∗ indicates statistical significant association.

**Table 4:** Seroprevalence of HCV with their sociodemographic characteristics and risk factors among pregnant women attending antenatal care at Borumeda General Hospital from April to May, 2020.

Variables	Categories	COR [95% CI]	*P* value	AOR [95% CI]	*P* value
Age (year)	15-25	1.00		—	—
	26 and above	0.451 (0.046-4.462)	0.496	—	—

Residence	Urban	1.00		—	—
	Rural	4.347 (0.439-43.023)	0.209	—	—

Marital status	Married	1.00		—	—
	Single	4.111 (0.387-43.668)	0.241	—	—

Educational status	Secondary & above	1.00		—	—
	Primary (1–8)	1.000 (0.059-17.015)	1.000	—	—
	Read & write	0.040 (0.026-7.358)	0.568	—	—
	Illiterate	0.846 (0.050-14.329)	0.908	—	—

Occupational status	Gov. employed	1.00		—	—
	Merchant	7.455 (0.435-127.891)	0.166	—	—
	Student	9.111 (0.524-158.455)	0.129	—	—
	House wife	4.556 (0.272-76.303)	0.292	—	—

Trimester	1^st^	1.00		—	—
	2^nd^	0.750 (0.045-12.436)	0.841	—	—
	3^rd^	01.535 (0.133-17.662)	0.731	—	—

Gravidity	Primigravida			—	—
	Multigravida	0.739 (0.101-5.424)	0.766	—	—

Previous place of delivery	No birth	1.00		—	—
	Health institution	0.625 (0.037-10.565)	0.745	—	—
	At home	0.588 (0.051-6.828)	0,671	—	—

Hospitalization with IV medication	Yes	2.167 (0.212-22.126)	0.514	—	—
	No	1.00		—	—

Surgical procedures	Yes	1.571 (0.156-15.857)	0.702	—	—
	No	1.00		—	—

Abortion history	Yes	8.231 (1.067-63.474)	0.043	7.991 (0.623-102.463)	0.110
	No	1.00			

History of blood transfusion	Yes	7.667 (0.672-87.421)	0.101	—	—
	No	1.00		—	—

Multi sexual partner	Yes	0.037 (0.004-0.385)	0.006	0.047 (0.001-2.861)	0.145
	No	1.00			

Condom usage	No	9.909 (1.268-77.413)	0.029	0.541 (0.013-21.765)	0.744
	Yes	1.00			

Sharing of sharp materials	Yes	2.070 (0.209-20.492)	0.534	—	—
	No	1.00		—	—

Ear and nose piercing	Yes	0.312 (0.032-3.083)	0.319	—	—
	No	1.00		—	—

Knife using in common	Yes	0.224 (0.030-1.682)	0.146	—	—
	No	1.00			

Drinking of alcohol	Yes	10.846 (1.083-108.666)	0.043	4.820 (0.284-81.780)	0.276
	No	1.00		1.00	

**Table 5:** Seroprevalence of HBV or HCV with their sociodemographic characteristics and risk factors among pregnant women attending antenatal care at Borumeda General Hospital from April to May, 2020.

Variables	Categories	COR [95% CI]	*P* value	AOR [95% CI]	*P* value
Age (year)	15-25	1.00			
	26 and above	0.745 (0.234-2.368)	0.617	—	—

Residence	Urban	1.00			
	Rural	1.444 (0.474-4.403)	0.518	—	—

Marital status	Married	1.00			
	Single	4.013 (0.906-17.780)	0.067	0.584 (0.024-14.205)	0.741

Educational status	Secondary & above	1.00			
	Primary (1–8)	2.211 (0.363-13.470)	0.390	—	—
	Read & write	0.894 (0.152-5.265)	0.901	—	—
	Illiterate	1.846 (0.303-11.020)	0.511	—	—

Occupational status	Gov. employed	1.00			
	Merchant	3.120 (0.53318.263)	0.207	2.031 (0.112-36.974)	0.632
	Student	6.686 (1.314-34.017)	0.022	8.811 (0.754-102.995)	0.083
	House wife	4.160 (0.999-17.317)	0.050	3.002 (0.269-33.548)	0.372

Trimester	3^rd^	1.00			
	2^nd^	0.388 (0.094-1.607)	0.192	1.332 (0.122-14.510)	0.814
	1^st^	0.724 (0.194-2.705)	0.631	0.851 (0.053-13.566)	0.909

Gravidity	Primigravida	1.00			
	Multigravida	1.926 (0.625-5.930)	0.253	1.112 (0.000-627.440)	0.983

Previous place of delivery	No birth	1.00			
	Health institution	0.586 (0.130-2.653)	0.488	-0.519 (0.044-6.177)	0.604
	At home	0.398 (0.101-1.574)	0.189	0.388 (0.00-6212.440)	0.848

Hospitalization with IV medication	Yes	6.750 (1.977-23.052)	0.002	6.214 (0.670-57.655)	0.108
	No	1.00			

Surgical procedures	Yes	3,039 (0.907-10.185)	0.072	0.486 (0.039-6.036)	0.575
	No	1.00			

Abortion history	Yes	8.417 (2.390-29.645)	0.001	11.069 (1.465-83.599)	0.020^∗∗^
	No	1.00			

History of blood transfusion	Yes	21.600 (3.511-132.888)	0.001	2.993 (0.089-101.137)	0.542
	No	1.00			

Multi sexual partner	Yes	0.051 (0.014-0.188)	0.001	0.000 (0.000...)	0.999
	No	1.00			

Condom usage	No	11.036 (2.989-40.750)	0.001	0.000 (0.000...)	0.999
	Yes	1.00			

Sharing of sharp materials	Yes	1.246 (0.392-3.965)	0.709	—	—
	No	1.00		—	—

Ear and nose piercing	Yes	1.500 (0.402-5.600)	0.546	—	—
	No	1.00			

Drinking of alcohol	Yes	4.000 (1.270-12.596)	0.018	1.164 (0.098-13.806)	0.904
	No	1.00			

∗∗ indicates statistical significant association.

## Data Availability

Those who want to find the original data that we have used for this study can get the data from the corresponding author with reasonable request.

## Abbreviations

HBV: Hepatitis B virus
HCV: Hepatitis C virus
WHO: World Health Organization
SOP: Standard Operating procedures (SOPs)
ANC: Antenatal clinic
IV: Intravenous.

## References

[1] Ndifontiayong A. N., Ali I. M., Sokoudjou J. B., Ndimumeh J. M., Tume C. B. (2021). The effect of HBV/HCV in response to HAART in HIV patients after 12 months in Kumba health district in the South West Region of Cameroon. *Tropical Medicine and Infectious Disease.*.

[2] Atlaw D., Sahiledengle B., Tariku Z. (2021). Hepatitis B and C virus infection among healthcare workers in Africa: a systematic review and meta-analysis. *Environmental Health and Preventive Medicine*.

[3] Coppola N., De Pascalis S., Onorato L., Calò F., Sagnelli C., Sagnelli E. (2016). Hepatitis B virus and hepatitis C virus infection in healthcare workers. *World journal of hepatology.*.

[4] Organization WH (2021). Global Progress Report on HIV, Viral Hepatitis and Sexually Transmitted Infections. *2021: Accountability for the Global Health Sector Strategies 2016–2021*.

[5] Hofstraat S., Falla A., Duffell E. (2017). Current prevalence of chronic hepatitis B and C virus infection in the general population, blood donors and pregnant women in the EU/EEA: a systematic review. *Epidemiology & Infection*.

[6] Geta M., Yizengaw E., Getaneh Z., Getahun T. (2021). Seroprevalence of hepatitis B virus infection among patients attending at Addis Alem Primary Hospital, Bahir Dar, Northwest Ethiopia. *International Journal of General Medicine.*.

[7] Elkhateeb R., Hassan K. (2018). Prevalence of hepatitis B and C in pregnant ladies and their neonates in Minia governorate. *International Journal of Pregnancy & Child Birth*.

[8] Fernandes C. N. S., Alves M. M., Souza M. L., Machado G. A., Couto G., Evangelista R. A. (2014). Prevalence of hepatitis B and C seropositivity in pregnant women. *Revista da Escola de Enfermagem da USP*.

[9] Dabsu R., Ejeta E. (2018). Seroepidemiology of hepatitis B and C virus infections among pregnant women attending antenatal clinic in selected health facilities in East Wollega Zone, West Oromia, Ethiopia. *BioMed Research International*.

[10] Zhao X., Bai X., Xi Y. (2022). Intrauterine infection and mother-to-child transmission of hepatitis B virus: route and molecular mechanism. *Infection and Drug Resistance.*.

[11] Umare A., Seyoum B., Gobena T., Haile M. T. (2016). Hepatitis B virus infections and associated factors among pregnant women attending antenatal care clinic at Deder Hospital, Eastern Ethiopia. *PLoS One*.

[12] Bancha B., Kinfe A. A., Chanko K. P., Workie S. B., Tadese T. (2020). Prevalence of hepatitis B viruses and associated factors among pregnant women attending antenatal clinics in public hospitals of Wolaita Zone, South Ethiopia. *Plo S one.*.

[13] Atalay A. A., Abebe R. K., Dadhi A. E., Bededa W. K. (2021). Seroprevalence of hepatitis B virus among pregnant women attending antenatal care in Dilla University Referral Hospital Gedio Zone, Ethiopia; health facility based cross-sectional study. *PLoS One*.

[14] Tanga A. T., Teshome M. A., Hiko D., Fikru C., Jilo G. K. (2019). Sero-prevalence of hepatitis B virus and associated factors among pregnant women in Gambella hospital, South Western Ethiopia: facility based cross-sectional study. *BMC Infectious Diseases*.

[15] Bafa T. A., Egata A. D. (2020). Seroepidemiological patterns and predictors of hepatitis B, C and HIV viruses among pregnant women attending antenatal care clinic of Atat Hospital. *SAGE Open Medicine*.

[16] Dessalegn Mekonnen B. (2021). Prevalence of hepatitis C virus infection among pregnant women in Ethiopia: a systematic review and meta-analysis. *Advances in Preventive Medicine*.

[17] Molla S., Munshea A., Nibret E. (2015). Seroprevalence of hepatitis B surface antigen and anti HCV antibody and its associated risk factors among pregnant women attending maternity ward of Felege Hiwot Referral Hospital, Northwest Ethiopia: a cross-sectional study. *Virology Journal*.

[18] Mamuye B., Gobena T., Oljira L. (2020). Hepatitis B virus infection and associated factors among pregnant women attending antenatal clinics in West Hararghe public hospitals, Oromia region, Ethiopia. *The Pan African Medical Journal*.

[19] Israr M., Ali F., Nawaz A. (2021). Seroepidemiology and associated risk factors of hepatitis B and C virus infections among pregnant women attending maternity wards at two hospitals in Swabi, Khyber Pakhtunkhwa, Pakistan. *PLoS One*.

[20] Wabe Y. A., Reda D. Y., Ali M. M. (2021). Seroprevalence of syphilis and HBV among pregnant women at Saint Paul s hospital millennium medical college, Addis Ababa Ethiopia. *Primary Health Care: Open Access*.

[21] Marama T., Shegaze M., Fikadu K. (2018). Burden of hepatitis B surface antigen sero-prevalence and associated factors among pregnant women receiving antenatal care at a public health institution, southern Ethiopia, 2018: implications for public health prevention. *Medical Studies/Studia Medyczne*.

[22] Desalegn Z., Mihret A., Beyene H. (2016). Survey of hepatitis B virus infection and risk factors among pregnant women at public hospital in Ethiopia. *International Journal of Biomedical Research*.

[23] Mudji J., Madinga B., Horsmans Y. (2021). Seroprevalence of viral hepatitis B and C and knowledge of the hepatitis B virus among pregnant women attending prenatal care in the Democratic Republic of Congo. *The American journal of tropical medicine and hygiene.*.

[24] Mac P., Suleiman A., Airiohuodion P. (2019). High prevalence of hepatitis B virus infection among pregnant women attending antenatal care in Central Nigeria. *Journal of Infectious Diseases and Epidemiology*.

[25] Taheu C. N., Nguwoh P. S., Demtaley A., Olinga P. Z., Fokam J. (2022). Seroprevalence of hepatitis B virus using HBV-5 rapid panel test and associated factors amongst pregnant women attending antenatal Care in Garoua, North-Cameroon. *European Journal of Medical and Health Sciences.*.

[26] Demeke G., Ayalneh G. M., Shiferaw A. A., Toru M., Dilnessa T. (2021). Sero-prevalence and associated factors of hepatitis B virus among pregnant women at north West Ethiopia: an institution-based cross-sectional study. *International Journal of General Medicine.*.

[27] Liu J., Wang X., Wang Q. (2021). Hepatitis B virus infection among 90 million pregnant women in 2853 Chinese counties, 2015-2020: a national observational study. *The Lancet Regional Health-Western Pacific*.

[28] Khattak S. T., Marwat M. A., Khan T. M., Naheed T. (2009). Comparison of frequency of hepatitis B and hepatitis C in pregnant women in urban and rural area of district Swat. *Journal of Ayub Medical College Abbottabad*.

[29] Dagnew M., Million Y., Gizachew M. (2020). Hepatitis B and C viruses’ infection and associated factors among pregnant women attending antenatal care in hospitals in the Amhara national regional state, Ethiopia. *International Journal of Microbiology*.

[30] Yohanes T., Zerdo Z., Chufamo N. (2016). Seroprevalence and predictors of hepatitis B virus infection among pregnant women attending routine antenatal care in Arba Minch Hospital, South Ethiopia. *Hepatitis Research and Treatment*.

[31] Nelson N. P., Easterbrook P. J., McMahon B. J. (2016). Epidemiology of hepatitis B virus infection and impact of vaccination on disease. *Clinics in Liver Disease*.

[32] Roble A. K., Roba K. T., Mengistie B., Kure M. A. (2020). Seroprevalence of hepatitis B virus and associated factors among pregnant women attending antenatal care in public health facilities in Jigjiga Town, Eastern Ethiopia. *International Journal of Women's Health*.

[33] Manyahi J., Msigwa Y., Mhimbira F., Majigo M. (2017). High sero-prevalence of hepatitis B virus and human immunodeficiency virus infections among pregnant women attending antenatal clinic at Temeke municipal health facilities, Dar es Salaam, Tanzania: a cross sectional study. *BMC Pregnancy and Childbirth*.

[34] Zenebe Y., Mulu W., Yimer M., Abera B. (2014). Sero-prevalence and risk factors of hepatitis B virus and human immunodeficiency virus infection among pregnant women in Bahir Dar city, Northwest Ethiopia: a cross sectional study. *BMC Infectious Diseases*.

[35] Musa B., Bussell S., Borodo M., Samaila A., Femi O. (2015). Prevalence of hepatitis B virus infection in Nigeria, 2000-2013: a systematic review and meta-analysis. *Nigerian Journal of Clinical Practice*.

[36] Geda Y. F., Desse H., Gesesse M. M., Berhe T. M. (2021). Hepatitis B surface antigen and associated factors among mothers who had antenatal care contact in Attat Hospital, southern Ethiopia. *SAGE Open Medicine*.

[37] Bayo P., Ochola E., Oleo C., Mwaka A. D. (2014). High prevalence of hepatitis B virus infection among pregnant women attending antenatal care: a cross-sectional study in two hospitals in northern Uganda. *BMJ Open*.

[38] Kirbak A. L. S. (2017). Sero-prevalence for hepatitis B virus among pregnant women attending antenatal clinic in Juba Teaching Hospital, Republic of South Sudan. *The Pan African Medical Journal*.

[39] Esan A., Omisakin C., Ojo-Bola T., Owoseni M., Fasakin K., Ogunleye A. (2014). Sero-prevalence of hepatitis B and hepatitis C virue co-infection among pregnant women in Nigeria. *American Journal of Biomedical Research*.

[40] Barros M. M. O., Ronchini K. R. O. M., Soares R. L. S. (2018). Hepatitis B and C in pregnant women attended by a prenatal program in an universitary hospital in Rio de Janeiro, Brazil: retrospective study of seroprevalence screening. *Arquivos de Gastroenterologia*.

[41] Makvandi M. (2016). Update on occult hepatitis B virus infection. *World journal of gastroenterology.*.

[42] Oti V., Mohammed I., Ibrahim Y., Ibrahim C., Orok I. (2021). Epidemiologic survey of HBV, HCV and HIV infections in a pregnant women population in Central Nigeria: a cross-sectional study. *Journal of Infectious Diseases and Epidemiology*.

[43] Ephraim R., Donko I., Sakyi S. A., Ampong J., Agbodjakey H. (2015). Seroprevalence and risk factors of hepatitis B and hepatitis C infections among pregnant women in the Asante Akim North Municipality of the Ashanti region, Ghana; a cross sectional study. *African health sciences.*.

[44] Oladeinde B. H., Omoregie R., Olley M., Anunibe J. A., Oladeinde O. B. (2012). Hepatitis B and C viral infections among pregnant women in a rural community of Nigeria. *International Journal of Basic and Applied Virology*.

[45] Omatola C. A., Lawal C., Omosayin D. O. (2019). Seroprevalence of HBV, HCV, and HIV and associated risk factors among apparently healthy pregnant women in Anyigba, Nigeria. *Viral Immunology*.

[46] Xiong H., Rong X., Wang M. (2017). HBV/HCV co-infection is associated with a high level of HCV spontaneous clearance among drug users and blood donors in China. *Journal of viral hepatitis.*.

[47] Tadiwos M. B., Kanno G. G., Areba A. S., Kabthymer R. H., Abate Z. G., Aregu M. B. (2021). Sero-prevalence of hepatitis B virus infection and associated factors among pregnant women attending antenatal care services in Gedeo Zone, Southern Ethiopia. *Journal of Primary Care & Community Health.*.

[48] Chernet A., Yesuf A., Alagaw A. (2017). Seroprevalence of hepatitis B virus surface antigen and factors associated among pregnant women in Dawuro zone, SNNPR, Southwest Ethiopia: a cross sectional study. *BMC Research Notes*.

[49] Amsalu A., Ferede G., Eshetie S., Tadewos A., Assegu D. (2018). Prevalence, infectivity, and associated risk factors of hepatitis B virus among pregnant women in Yirgalem hospital, Ethiopia: implication of screening to control mother-to-child transmission. *Journal of Pregnancy*.

[50] Mulu W., Zenebe Y., Abera B., Yimer M., Hailu T. (2016). Prevalence of human immunodeficiency virus and hepatitis B virus infections in young women seeking abortion care in Ethiopia: a cross - sectional study. *BMC Public Health*.

[51] Hervish A., Clifton D., UNFPA (2012). *Status report: adolescents and young people in Sub-Saharan Africa*.

[52] Moore A. M., Gebrehiwot Y., Fetters T. (2016). The estimated incidence of induced abortion in Ethiopia, 2014: changes in the provision of services since 2008. *International perspectives on sexual and reproductive health.*.

[53] Tesfaye G., Hambisa M. T., Semahegn A. (2014). Induced abortion and associated factors in health facilities of Guraghe zone, southern Ethiopia. *Journal of Pregnancy*.

[54] River T., Jersey N. (2014). Sexually transmitted infections. *The Healthy Woman A Complete Guide For All Ages*.

[55] Farshadpour F., Taherkhani R., Bakhtiari F. (2021). Prevalence and predominant genotype of hepatitis C virus infection and associated risk factors among pregnant women in Iran. *BioMed Research International*.

[56] Mostafa A., Ebeid F. S., Khaled B., Ahmed R. H., El-Sayed M. H. (2020). Micro-elimination of hepatitis C through testing of Egyptian pregnant women presenting at delivery: implications for screening policies. *Tropical Medicine & International Health*.

